The article "Estimation of the Serial Interval and the Effective Reproductive Number of COVID-19 Outbreak Using Contact Data in Burkina Faso, a Sub-Saharan African Country" was published in 2022. Journal: Comput Math Methods Med.

# Estimation of the Serial Interval and the Effective Reproductive Number of COVID-19 Outbreak Using Contact Data in Burkina Faso, a Sub-Saharan African Country

**DOI:** 10.1155/2022/8239915

**Published:** 2022-09-25

**Authors:** Serge M. A. Somda, Boukary Ouedraogo, Constant B. Pare, Seni Kouanda

**Affiliations:** ^1^UFR-Sciences Exactes et Appliquées, Université Nazi Boni, Bobo-Dioulasso, Burkina Faso; ^2^Centre Muraz, Institut National de Santé Publique (INSP), Bobo-Dioulasso, Burkina Faso; ^3^Direction des Systèmes d'Information en Santè (DSIS), Ministère de la Santé, Ouagadougou, Burkina Faso; ^4^Département de Sante Publique, Unité de Formation et de Recherche en Sciences de la Sante Université Joseph Ki-Zerbo, Ouagadougou, Burkina Faso; ^5^Institut de Recherche en Sciences de la Santé (IRSS), Ouagadougou, Burkina Faso; ^6^Institut Africain de Santé Publique (IASP), Ouagadougou, Burkina Faso

## Abstract

The COVID-19 outbreak has spread all around the world in less than four months. However, the pattern of the epidemic was different according to the countries. We propose this paper to describe the transmission network and to estimate the serial interval and the reproductive number of the novel coronavirus disease (COVID-19) in Burkina Faso, a Sub-Saharan African country. Data from the COVID-19 response team was analyzed. Information on the 804 first detected cases were pulled together. From contact tracing information, 126 infector-infectee pairs were built. The principal infection clusters with their index cases were observed, principally the two major identified indexes in Burkina. However, the generations of infections were usually short (less than four). The serial interval was estimated to follow a gamma distribution with a shape parameter 1.04 (95% credibility interval: 0.69–1.57) and a scale parameter of 5.69 (95% credibility interval: 3.76–9.11). The basic reproductive number was estimated at 2.36 (95% confidence interval: 1.46–3.26). However, the effective reproductive number decreases very quickly, reaching a minimum value of 0.20 (95% confidence interval: 0.06–0.34). Estimated parameters are made available to monitor the outbreak in Sub-Saharan African countries. These show serial intervals like in the other continents but less infectiousness.

## 1. Introduction

The COVID-19 outbreak has appeared in Wuhan city, Hubei district in December 2019 [1]. The number of cases rapidly expands through the country and beyond. This disease was declared Public Health Emergency of International Concern (PHEIC) by the Director General of the World Health Organization (WHO) on January 31, 2020, and finally considered as a pandemic in March 2021 [2]. The spread of the epidemic was found exceptionally high. At the reference date of data collection, no drug or vaccine was validated. It was therefore urging to forecast the spread and the probable size, in terms of space and time to propose effective measures to mitigate or to stop the situation.

Very early mathematical studies were undergone to understand the spread of the disease. The absolute first ones principally consist in susceptible-infectious-recovered models. Farman et al. analyzed the equilibrium point and the stability of such models [3] applied to the disease. However, all these needed to feed from strong assumptions in the absence of evidence from the field. This evidence was made available for some countries. Lai et al. [4] proposed very early, in February 2020, an estimation of the reproductive number, using phylogenetic analysis. They could benefit of 52 SARS-CoV-2 sequences which, after analysis, could permit to say that the epidemic was presenting a mean effective reproductive number of 0.8 at its beginning which evolved to 2.6 in February. Li et al. [5] used patient tracing data and found a mean serial interval of 7.4 days and a basic reproductive number of 2.2, based on six infector-infectee pairs. Nishiura et al. [6] then had access to 28 pairs and could find a median serial interval of 4.6 days. Other data driven estimations can be found for the Diamond Princess cruise ship [7], in Shenzhen (K. [8]) and in Hong Kong (Zhao et al., [9]). Estimations of the reproductive number can also be found for European [10] and American [11] countries.

The first COVID-19 case in Sub Saharan Africa (SSA) was declared in Nigeria the 27^th^ February 2020 [12]. All the governments and regional institutions were then mobilized on the continent to stop the spread of the pandemic. The strategies undergone in Asia and in Europe few months ago were adapted and applied. However, all the specialists admitted that the pandemic does not have the same characteristic in Africa. They then considered that it will not be efficient to plan for the spread of the disease based on the Asian or European estimations of the diseases spread characteristics. To our knowledge, there is no publication on the estimates of the reproductive number in Sub–Saharan Africa. Early-stage modeling activities can be found in Burkina Faso. The approach of SIR models with more compartments was proposed by Guiro et al. who could bring the first estimates on the epidemic in Burkina Faso [13]. Konane and Traore proposed a fast forecasting approach but this was a pure time series analysis using ARIMA methods [14]. Other studies could model and predict the effect of public health interventions in the early stages [15]. However, none could really describe the serial interval and the effective reproductive number based on that kind of detailed data. Our objective is to produce estimates of both the serial interval and the reproductive number in Burkina Faso, a West African country, using a standardized method which can be easily reproduced for other epidemics.

## 2. Material and Methods

### 2.1. Study Setting and Type of Study

This a secondary analysis of the data of COVID-19 collected routinely in the Integrated Disease Surveillance and Response (IDSR) team and by Centre des Opérations et de Réponse aux Urgences Sanitaires (CORUS), within the National of Public Health Institute during the early period of the outbreak in Burkina Faso.

Burkina Faso is a landlocked Sahelian country in the heart of West Africa. It has an area of around 270,200 square kilometers. The country is divided into 13 regions, 45 provinces, and 351 municipalities. The population was estimated at 21,510,181 inhabitants in 2020 according to the national statistics institute. The majority of the population lives in rural areas, with agriculture and livestock as main activities in 2019.

Burkina recorded their first two COVID-19 cases on March 9, 2020. Then, as of March 31, 2020, 282 confirmed cases were identified in height regions out of the 13 in the country. On May 21^st^, 812 confirmed cases were observed. Among them, 669 were recovered and unfortunately 52 died. The case fatality ratio (CFR) was 6.42%.

At this same moment, the World Health Organization (WHO) was reporting 4,893,186 cases with a CFR of 6.61% globally. The African Region was counting 68,347 cases with a CFR of 2.79%. Africa has the lowest CFR among the six WHO regions. Burkina Faso unfortunately was presenting a CFR among the higher in the continent and particularly the third higher in the ECOWAS region after Liberia (9.58%) and Niger (6.49%).

### 2.2. Concepts and Definitions

The serial interval is defined as the time interval between symptom onset of an infector and symptom onset of its infectee [16]. This is slightly different from the generation time which is defined as the interval between a case becoming infected and its subsequent infection of another case [16, 17]. Each time interval *u* between the infection time of a primary and a secondary case is considered as generated from a probability distribution function *ϖ*(*u*, Θ) with parameter(s) Θ [18].

Reich et al. [19] proposed an approach to estimate incubation period using doubly interval-censored data. For example, for Gamma distributed intervals, assuming parameters Θ = (*θ*, *k*), the likelihood is defined as follows:

(1) $$\begin{array}{c} \varpi \left(u,\theta ,\text{k}\right)=\frac{1}{\theta^{k}\Gamma \left(u\right)}u^{k-1}e^{-u/\theta }. \end{array}$$

The reproductive number is a key indicator for monitoring and for prediction of epidemics. This is a key value to model infectious diseases either using differential equations or statistical approaches. It can be defined as the average of secondary cases of disease caused by a single infected individual over his or her infectious period. As an example, we propose here two approaches to define the effective reproductive number.

The first is based on a standard susceptible-infectious-removed (SIR) model with:

(2) $$\begin{array}{c} \frac{dS}{dt}=-\beta \frac{S}{N}I;\frac{dI}{dt}=\beta \frac{S}{N}I-\gamma I, \end{array}$$

where *S*(*t*), *I*(*t*), and *N*(*t*) are, respectively, the average number of susceptible, the average number of infectious, and the size of the population at time *t*. *β* is the contact rate, and 1/*γ* is the average infectious period. The basic reproductive number, *R*_0_, is the statistic usually estimated and defined as the expected number of secondary cases produced by a single (typical) infection in a completely susceptible population. It can be defined as [20]

(3) $$\begin{array}{c} R_{0}=\frac{\beta }{\gamma }. \end{array}$$

This equation assumes that the reproductive number is constant over time and that the infectiousness is exponentially distributed. In this case, an “instantaneous reproductive” number can be defined as *R*_*t*_ = *β*(*S*(*t*)/*N*(*t*))*R*_0_. Then, the number of infectious cases to come after a duration *s* is approximated as [20]

(4) $$\begin{array}{c} I\left(t+s\right)=I\left(t\right)e^{s\gamma \left(R_{t}-1\right)}. \end{array}$$

However, the reproductive number is time and situation specific. Then, the concept of effective reproductive number is also used. The effective reproductive *R*_*t*_ number is defined roughly as the average number of people someone infected at time *t* can infect over their entire infectious lifespan [21]. Several approaches of estimation of the effective reproductive number using surveillance data can be found in literature [20–23].

Cori et al. assumed that the distribution of infectiousness through time after infection is independent of calendar time [21, 24]. This second approach is using a renewal process. They model the transmission with a Poisson process was an individual infected at time *t* − *s* will generate new infections at time *t* with a rate *R*_*t*_*w*_*s*_, where *R*_*t*_ is the instantaneous reproduction number at time *t* and *w*_*s*_ the infectiousness profile. Considering *I*_*t*_ the incidence at time *t*, *Λ*_*t*_ = ∑_*s*=1_^*t*^*I*_*t*−*s*_*w*_*s*_ can be considered as the average number of infected cases between the time *t* − *s* and *t*. The likelihood of the incidence *I*_*t*_ given the reproduction number *R*_*t*_ conditional on the previous incidences *I*_0_, ⋯, *I*_*t*−1_ is

(5) $$\begin{array}{c} P\left(I_{t}\left|I_{t-1},\cdots ,I_{0},R_{t}\right.\right)=\frac{{\left(R_{t}\;\Lambda_{t}\right)}^{I_{t}\;e^{-R_{t}\;\Lambda_{t}}}}{I_{t}!}. \end{array}$$

While modeling, the local infectious cases should be separated from the imported ones. In fact, even though the later contribute to the new infections, they are not part of the estimators. Considering *L*_*t*_ and *M*_*t*_ as the number of local and imported new infectious cases at time *t* with *L*_*t*_ + *M*_*t*_ = *I*_*t*_, the likelihood of the local incident cases *L*_*t*_ according to all the historical cases is

(6) $$\begin{array}{c} P\left(L_{t}\left|L_{t-1},\cdots ,L_{0},M_{t-1},\cdots ,M_{0},R_{t}\right.\right)=\frac{{\left(R_{t}\;\Lambda_{t}\right)}^{L_{t}\;e^{-R_{t}\;\Lambda_{t}}}}{L_{t}!}. \end{array}$$

Assuming a constant transmissibility over a time period [*t* − *τ* + 1; *t*] where the reproductive number is noted *R*_*t*,*τ*_, this indicator is defined with Gamma distributed prior parameters (*a*, *b*), and the posterior distribution is a Gamma distribution with parameters:

(7) $$\begin{array}{c} \left(a+\overset{t}{\underset{s=t-\tau +1}{\sum }}I_{s},\frac{1}{1/b+\sum_{s=t-\tau +1}^{t}\Lambda_{s}}\right). \end{array}$$

In this case, the posterior mean and posterior standard deviation of *R*_*t*,*τ*_ are, respectively

(8) $$\begin{array}{c} \frac{a+\sum_{s=t-\tau +1}^{t}I_{s}}{1/b+\sum_{s=t-\tau +1}^{t}\Lambda_{s}}\text{ and }\frac{\sqrt{a+\sum_{s=t-\tau +1}^{t}I_{s}}}{1/b+\sum_{s=t-\tau +1}^{t}\Lambda_{s}}. \end{array}$$

### 2.3. Data Sources

The surveillance system of the COVID-19 outbreak in Burkina Faso is organized as follows: (1) warning data which are information on people calling the emergency number for COVID-19 investigation, (2) contact tracing data, (3) entry point data, (4) rapid response team's data, (5) laboratory data, and (6) case management data. All these are stored and managed into a DHIS2 platform in the Ministry of Health. The staff have been granted tablets for fast and remote updates of the platform.

Three datasets were used for the analysis. The data on confirmed cases (804 records), the data on contact tracing (4,523 records), and the data on infector-infectee follow-up which relate each case to the probable case who infected him (113 records). The data were fed from the date of confirmation of the first case (9 March 2020) to the 21 May 2020.

### 2.4. Data Analysis

A first curation process was applied to the data. The duplicate information and the inconsistencies were cleared. The different data tables have also to be conciliated and the pairs made consistent.

The network analysis was performed using *ggraph* package [25] in R. The *EpiEstim* package [24, 26] was used for the epidemic parameters estimation. This uses a two-step procedure to estimate the effective reproductive number from data informing the serial interval and from data on the incidence of cases over time [27]. The approach consists in a Bayesian parametric estimation of the serial interval distribution from the time data between infector and infectee using Monte Carlo Markov Chains (MCMC). The *coarseDataTools* package [28] is used to fit the serial interval distribution. The reproductive number was computed using inference with MCMC chains where imported cases were distinguished from local transmissions. In fact, imported cases are contributing to the expansion of the transmission like local ones. However, they are not consequences of the previous state of the epidemic unlike local cases. The renewal process approach to estimate the reproductive number is the one implemented in this paper.

Some sensitivity analyses were performed by Cori et al. when presenting their method. The estimation of the reproductive number has been described as sensitive to the time window. Strategies were then proposed to have optimal windows. The estimations are also extremely sensitive to the time steps. Then, the package proposes as default daily records. The quality of the estimation was assessed by simulation [24].

The serial interval was simulated considering the date of sample taking for laboratory testing. The recommended variable is the date of symptom onset but this one was not available in the database. However, a simulation analysis performed by Cori et al. [24] showed that the use of date of symptom onset do not create any bias in the estimations. A parametric gamma distribution was then fitted [19, 28]. The number of burning replications was set to 3000 with a thin count of 10. Then, 5000 serial interval distributions were generated, and samples of size 500 were drawn from the posterior distribution.

We have processed the data and removed duplicate observations. To facilitate data visualization, a loess smoothing was applied on the median effective reproductive number.

## 3. Results

### 3.1. Sample Description

Data on 804 cases were analyzed including 499 (62.06%) male, 300 (37.31%) female, and 5 without information on gender. The median age was 42 years (IQR = 30–57). This was 42 years (IQR = 29–58) for men and 43 years (IQR = 32–56) for women. The distribution by dates shows that the cases were increasing very fast at the beginning (day 0 to day 30) and then had a slow decrease (day 30 to day 73). In 73 days of the epidemic, two major modes could be identified in the distribution in March 2020 and in April 2020 plus a minor one early in May (Figure 1). These peaks correspond to slight differences in gender distribution where women were infected generally later than men.

### 3.2. Network Analysis

The contact tracing data could record 142 infectors-infectee transmission. However, after checking, 16 observations were removed as duplicates. Then, 126 unique pairs were analyzed.

The plotted network could reveal four principal clusters with three generations and more than five secondary cases (Figure 2). The two largest clusters' index cases were famous personalities who were in contact with several people at their return from Europe. One can notice that the maximum number of generations observed was three. This means that after 73 days, we could not have evidence of any fourth generation of case. However, some infection cases were related to two infectors in the data. This means that the case was in contact with two known infected cases.

### 3.3. Serial Interval and Reproductive Number

Figure 3 presents the distribution of time between the date the infector was confirmed for COVID-19 and the date when the infectee was. The first infector was confirmed on March 9^th^ as the latest in the dataset was on April 1^st^. The infectees were confirmed in both March and April ranging from March 12^th^ to April 21^st^. The Figure 3 shows that the infectious time was very variable from one case to another and that this could reach three weeks. The largest timespan between the time the infector was confirmed, and the time the infectee was confirmed was 30 days. The median value was 5 days (interquartile range 1 to 10 days). Negative timespans were found for 5 cases (-7 to -4) while 21 infector-infectee pairs were confirmed the same day.

The gamma distribution corresponding to the serial interval had an estimated shape parameter of 1.04 (95% credibility interval: 0.69–1.57) and an estimated scale parameter of 5.69 (95% credibility interval: 3.76–9.11). The median value was 4.20 (95% credibility interval: 3.03–5.37). The distribution was simulated and presented in Figure 4, with the raw data presented in dashed histogram. The estimated mean distribution is 3.91 with a standard deviation of 3.81.

The simulated mean effective reproductive number was estimated at 2.36 (95% confidence interval: 1.46–3.26), at the beginning of the epidemic (Figure 5). This means that the first index cases infected around two to three people. However, the effective reproductive number decreased very quickly. It reached one in around ten days. Since the latest week of March, the effective number was under one. The estimated smallest estimated mean was 0.20 (95% confidence interval: 0.06–0.34). Unfortunately, the estimation shows an increase after this minimum value.

Since the onset of the disease in March, our analysis shows a decrease in the reproductive number which was more significant in early March. The estimated value decreased sharply under one (1) on March 21 with a low on March 28. We found a slight rebound after this last date but still very low (under one).

## 4. Discussion

This is a first estimation of reproductive number and serial interval in Sub-Saharan Africa. The COVID-19 epidemic is characterized by the lack of epidemiological information. The absence of these estimations is more pronounced in Sub-Saharan Africa. Even in the most recent publications on the outbreak in the region [29–31], the model parameters were obtained from studies outside the region.

Our estimations provided an effective reproductive number from 2.33 at the beginning of the epidemic. However, this figure declined very rapidly, meaning that transmission was becoming lower and lower. This could be explained by several factors. The first factor is the low detection rate at the beginning of the pandemic (in fact only one reference laboratory was testing for one month at during this period); the second one is the strong governmental actions two weeks after the first case specifically the distancing measures, the quarantine, the use of hydroalcoholic gel, the wearing of masks, the closure of schools, high schools, and universities, and the closure of markets and international borders.

The negative values observed for time between the infection of the infector and the infection of the infectee are not implausible. Due to the large variability among people susceptible to be infected, the observed incubation periods are also highly variable. This can lead to this situation, which has already been described elsewhere [6]. This also gives credit of the hypothesis of asymptomatic transmission and even presymptomatic transmission. The value used to estimate serial interval is usually the date of symptoms onset. This data was unfortunately not available. We used the date of confirmation instead as generally the tracked contacts were tested immediately when they declare to have symptoms. The approach used to estimate the reproductive number considers that infectiousness only starts at or after the time of symptom onset. This may be a bias in our estimation. However, the negative values observed are very low in term of number and can be neglected.

The estimated distribution of the serial interval presents a shape parameter which is not significantly different to 1 (1.04 with 95% credibility interval: 0.69–1.57). This is likely to be an exponential distribution. Then, we can state that the hazard of transmitting the infection is constant once an individual is infected. The values of serial interval from our analysis are 4.20 (95% credibility interval: 3.03–5.37) days. Nishiura et al. estimated the median to 4.6 days [6]. Wang et al. (K. [8]) used the same gamma approach and had also a median of 4.8 days. Then, several authors found more than 5 days ([32]; Ganyani et al., [33]; [5]). Additionally, the mean and median serial interval is smaller than the described incubation time [5, 34, 35] which is around 5 days. The reproductive number is hard to compare with the literature as the patterns are generally presented into different ways. However, it will be recommended to work on estimations which are geographically closer to mitigate the eventual effect of other factors (e.g., climate).

The contact tracing and the surveillance data showed several cases which could not be relied to an infector. This highlights the fact that they may be several asymptomatic carriers in the population. The World Health Organization indicated that 80% of the infections are mild or asymptomatic [36]. However, nonpublished information in some Sub-Saharan African countries estimated that 77 to 86% of the cases were asymptomatic. This highlights the need of a general prevalence survey in the region. The data also revealed sometimes more than one probable infector for a case. This states that there may be inaccuracy in the identification of the infector. A wide phylogenic study could permit a mapping of the infection trend and to build a comprehensive tree. This will also help to understand the transmission pattern in our countries and increase the preparedness for upcoming health problems.

Finally, fourth generation of infection was never observed. This shows a good contact tracing procedure in the country. All the clusters were killed very soon so that no massive spread was observed. This can be one good reason why there are relatively very few cases in Burkina Faso so far. To our knowledge, the network presented on Figure 2 is the first for a Sub-Saharan country since the apparition of COVID-19 pandemic in the continent. Tindale et al. [37] presented the network for Singapore and Tianjin (China) in early 2020, and this was presenting the same pattern. There were no long descendance in terms of history of infection. Like Wang and Teunis (Y. [38]), in their study in Tianjin, China, the network shows that imported cases created important clusters. This is to say that some individual cases could have spread the disease to many people.

The presented study has some limitations which need to be highlighted. The gamma distribution is the most frequently used to estimate serial interval ([5, 16, 21, 24]; Zhao et al., [9]). This distribution is very flexible and suitable for several contexts. However, the gamma distribution only suits for positive values. Then, the proposed model cannot generate negative serial intervals. The data which were used presented many flaws. Discussions are still ongoing on the capacity of the system to detect cases. Many authors highlighted the fact that the countries are not able to detect most of the COVID-19 cases. Not yet published seroprevalence surveys that were run in the region should confirm the large number of missed COVID-19 cases [39]. In line with the capacity to detect the cases, the capacity to track contacts and to properly associate infectors and infectees was also a big concern.

We did not have enough data to discuss on the effect of public measures such as case isolation. All cases were isolated starting at their data of confirmation. However, no data exists on the infectiousness before and after the isolation, as the date of infection was not available.

However, the study presents strengths which should be emphasized. The methodology to determine both the serial interval and the reproductive number is rigorous and widely validated. This relies on strong probabilistic background and has been used widely, principally to estimate COVID-19 parameters.

Our estimations of the key parameters of COVID-19 pandemic in Burkina Faso can be considered as quite obsolete. In fact, several epidemic waves of the disease have been observed since May 2020, implying new distributions for the estimated values. These are probably due to significant changes in the context of the disease (individual behaviors and implementation of public health measures). Additionally, several variants of interest have been observed for the COVID-19 disease. The recent models now consider quarantine and social distancing [40, 41], weather [42], epidemic waves [43, 44], or vaccination [40, 45]. The presented results are still of high importance as these observed primary characteristics can be used to propose a better follow-up and understanding of the disease spread in Burkina Faso as well as in other African countries. More recent approaches [46] will be adapted to this information to take into account the new observed patterns. It is also crucial for next preparation to know the real situation of the outbreak in our countries and to compare it with the different assumptions the researchers and decision makers had to make in the total absence of local reliable estimations. This knowledge will guide for possible upcoming public health emergencies.

Two years and a half after the apparition of the disease, the world has experienced several epidemic phases, which were called waves. These waves are attributed to seasons and the apparition of several variants of concern [42, 47, 48]. Even though the definition of these waves is not clear, the West African region is considered to have passed through four major ones. Meanwhile, Burkina Faso has had his two major waves from December 2020 to February 2021 and in January 2022. The country is reporting as of July 17, 2022, a total of 21,128 confirmed cases and 387 deaths, according to the West African Health Organization. This was 2.5% of the cases in the ECOWAS region. The authors proposed models through all these waves [42, 49]. However, we found it useful to insist on the absolute early moment of the introduction of the disease where the trend is not due to multiple factors yet. Modeling the epidemic now will require the consideration of several aspects which occurred with time and which could hardly be associated to another epidemic. Then, the quality of the data, and particularly, of the contact tracing is decreasing as the number of cases and the fatigue of the response teams are increasing. Even though we are rising concerns on the quality of the data we used, we are sure that such quality data cannot be obtained if we extend to one year or more.

Meanwhile, several modeling exercises were proposed to better understand the pandemic in our region. Ayinde et al. [50] found it useful to use a quartic curve estimation model to forecast the epidemiological parameters in West African countries.

The underreporting of COVID-19 cases has been a big challenge for the response to the pandemic, particularly in Africa. As the testing rate was insufficient, it is expected that several cases have not been detected nor confirmed. This is a major issue in any statistical or epidemiological analysis on COVID-19. However, Cori et al. described their approach as being robust to underreporting even though the estimators may have more variability [24]. Our study relied only on reported data. As we are publishing these results, we believe that the transmission rates can be higher. However, as an exercise, it demonstrates the use of the data to find the relevant parameters to inform decision making and provide targeted results.

## Figures and Tables

**Figure 1:** Distribution of the COVID-19 infection dates by gender in Burkina Faso.

**Figure 2:** COVID-19 infection network in Burkina Faso.

**Figure 3:** Infector-infectee dates of confirmation the COVID-19 infection.

**Figure 4:** Density distribution of the estimated COVID-19 outbreak serial interval in Burkina Faso, raw data are presented in dashed histograms.

**Figure 5:** Effective reproductive number for the early COVID-19 outbreak in Burkina Faso.

## Data Availability

The used data were collected and managed by the Centre des Opérations et de Réponse aux Urgences Sanitaires (CORUS), within the National Public Health Institute in Burkina. The data is available through formal request to secretariat@insp.gov.bf.
